This article has been retracted.

# Computational Insights into the Structural and Functional Impacts of nsSNPs of Bone Morphogenetic Proteins

**DOI:** 10.1155/2022/4013729

**Published:** 2022-07-04

**Authors:** Hafiz Ishfaq Ahmad, Nabeel Ijaz, Gulnaz Afzal, Akhtar Rasool Asif, Aziz ur Rehman, Abdur Rahman, Irfan Ahmed, Muhammad Yousaf, Abdelmotaleb Elokil, Sayyed Aun Muhammad, Sarah M. Albogami, Saqer S. Alotaibi

**Affiliations:** ^1^Department of Animal Breeding and Genetics, University of Veterinary and Animal Sciences, Lahore, Pakistan; ^2^Department of Clinical Science, Faculty of Veterinary Sciences, Bahauddin Zakariya University Multan, Pakistan; ^3^Department of Zoology, The Islamia University of Bahawalpur, Bahawalpur, Pakistan; ^4^Key Laboratory of Animal Genetics, Breeding and Reproduction, Huazhong Agricultural University, Wuhan, China; ^5^University of Veterinary and Animal Sciences, Lahore, Sub-Campus Jhang, Pakistan; ^6^Department of Animal Nutrition, Afyon Kocatepe University, Turkey; ^7^Department of Animal Nutrition, Faculty of Veterinary and Animal Sciences, The Islamia University of Bahawalpur, Pakistan; ^8^Department of Animal Production, Faculty of Agriculture, Benha University, Moshtohor 13736, Egypt; ^9^Department of Biotechnology, College of Science, Taif University, P.O. Box 11099, Taif 21944, Saudi Arabia

## Abstract

BMPs (bone morphogenetic proteins) are multipurpose (transforming growth factor)TGF-superfamily released cytokines. These glycoproteins, acting as disulfide-linked homo- or heterodimers, are highly potent regulators of bone and cartilage production and repair, cell proliferation throughout embryonic development, and bone homeostasis in the adults. Due to the fact that genetic variation might influence structural functions, this study is aimed to determine the pathogenic effect of nonsynonymous single-nucleotide polymorphisms (nsSNPs) in BMP genes. The implications of these variations, investigated using computational analysis and molecular models of the mature TGF-*β* domain, revealed the impact of modifications on the function of BMP protein. The three-dimensional (3D) structure analysis was performed on the nsSNP Y316S, V386G, E387G, C389G, and C391G nsSNP in the TGF-*β* domain of chicken BMP2 and H344P, S347P, V357A nsSNP in the TGF-*β* domain of chicken BMP4 protein that was anticipated to be harmful and of high risk. The ability of the proteins to perform variety of tasks interact with other molecules depends on their tertiary structural composition. The current analysis revealed the four most damaging variants (Y316S, V386G, E387G, C389G, and C391G), highly conserved and functional and are located in the TGF-beta domain of BMP2 and BMP4. The amino acid substitutions E387G, C389G, and C391G are discovered in the binding region. It was observed that the mutations in the TGF-beta domain caused significant changes in its structural organization including the substrate binding sites. Current findings will assist future research focused on the role of these variants in BMP function loss and their role in skeletal disorders, and this will possibly help to develop practical strategies for treating bone-related conditions.

## 1. Introduction

Bone mineralization involves preosteoblastic cells, physicochemical reactions, and an organic matrix framework [1]. Plasma and extracellular fluids include various calcium and phosphate ions which regulates and nucleate the deposition of hydroxyapatite crystals in the gap between collagen molecules [2]. Bone defect repair is an ideal model for studying bone regeneration because reparative regeneration happens due to accidents or illnesses. Abrasions are far less sensitive to mechanical forces and are less susceptible to obstructions in the circulatory system [3]. Preosteoblastic cells were active in the regeneration of rabbit tibia bone defects. It was discovered that bone development was initiated within a few days without osteoclastic bone adherence [4]. Skeletal abnormalities are observed more frequently in the broilers that usually grow rapidly and are less active. In general, the absence of necessary activity leads to an increase in skeletal disorders among the birds [5].

Additionally, researchers found that the size of the defect, the function of pre-osteogenic cells, and the mechanisms that regulate their growth, maturation, and process all had an impact on bone regeneration [6]. The migration and division of mesenchymal stem cells (MSCs), as well as their differentiation and maturation into osteoprogenitor cells and osteocytes, are the defining characteristics of the process known as osteogenesis [7]. BMPs have a role in bone and cartilage growth and also in mature bone function homeostasis, although BMPs were recognized as to encourage bone development [8]. Furthermore, deletion of BMP7 from the embryonic limb in mice had no effect [9]. BMP7 deficient mice, on the other hand, have rib, skull, and hind limb skeletal patterning abnormalities [10]. BMP11 is also involved in the skeletal patterning throughout the development BMP11 mutants that have been observed to alter the expression of HOX gene and caused abnormal axial skeleton [11].

The growth differentiation factor (GDF 5) plays a significant role in bone and joint development [12]. BMP13 mutations have been reported to cause developmental issues at various body locations, including the wrist and ankle. BMP13 knockout mice fused coronal sutures quicker, showing that BMP13 suppresses osteogenic differentiation [13]. The junction of the carpal and tarsal bones also identifies BMP13 mutations. An in vitro study confirmed that this BMP has a robust inhibitory effect [14]. The involvement of BMP in tendon biology was discovered by studying the phenotypic of the tendon in mice carrying BMP mutations [15].

Osteoblast abnormalities include brittleness, spontaneous fractures, disturbed fracture healing, scoliosis, kyphosis, developmental ossification, postnatal skeletal overgrowth at non-skeletal locations periosteal growth, changed quantity of bone mass, and an aberrant quality of bone matrix. There are several types of chondrodysplasia chondrodysplastic disease, dwarfism, unusual long-term growth (brachypodism), faulty or accelerated chondrogenesis, and problems in the cartilage template vascularization [16]. Failure to establish synovial or nonsynovial joints during the development and issues related to the production of mature joint structures such as the meniscus, tendons, ligaments, and osteoarthritis are all examples of joint abnormalities [17]. Tibial dyschondroplasia (TD) is another bone disorder with several underlying causes such as uncoupling of growth plate chondrocyte proliferation and endochondral ossification during bone elongation [18]. As a result, mass of uncalcified cartilage forms at the proximal end of long bones (primarily the tibiotarsus, but not exclusively). Further research is still required to elucidate the cellular and molecular mechanisms behind the bone elongation and to narrow down the other possible causes of this skeletal anomaly [19].

A study examined the walking abilities (gait scores) of traditional broilers and discovered that 77.4 per cent of birds had an irregular gait, with 5.5 percent having significant gait impairments (gait score 2). Besides that, 4.7 percent of the broilers were found to have tibial dyschondroplasia, and 6.5 percent were found to have inflammation of the hock joint tendon sheath (tenosynovitis) [20]. Lameness was shown to be associated with both of these diseases. Skeletal abnormalities create persistent discomfort making it harder for the broilers to obtain food and water, thus significantly impacting their health and overall performance [21]. Broilers that have been affected by this disease are unable to get up quickly and end up lying on the floor until they die from dehydration (Julian 1998). In commercial broilers, non-infectious skeletal illnesses including articular gout, degenerative joint disease, dyschondroplasia, rickets, rotational angular deformities, spondylopathies, and ruptured gastrocnemius tendon have been reported among others.

This work examined possible detrimental SNPs in the BMP2 and BMP4 genes of chicken, which might impair the protein's structural and dynamic integrity. This study is aimed to study the role of BMP in skeletal development and to find a series of missense mutations in chickens. The appearance of these variations, investigated using computational analysis and molecular models of the mature TGF-beta domain, revealed how the mutations might impact BMP protein function. The current study showed that GDF3 plays a crucial and evolutionarily role in the skeletal development and new multi-allelic inheritance of BMP variations in developmental illness.

## 2. Materials and Methods

### 2.1. Data Collection

The SNP data for the BMP genes were obtained from the National Center for Biotechnology Information, USA (NCBI) dbSNP (http://www.ncbi.nlm.nih.gov/snp/), and Ensembl database (http://asia.ensembl.org/Gallus gallus/Gene/Variation Gene/). Each SNP has its unique reference sequence ID (rsID) (supplementary file). BMP genes' amino acid sequence and the BMP genes' sequence were obtained from the UniProt database (Q90751 and Q90752). BMP genes' sequence was also obtained from the National Center for Biotechnology Information (NCBI) (http://www.ncbi.nlm.nih.gov/gene/). This information used for further computational analysis.

### 2.2. Detection of Harmful SNPs

The SNP database (dbSNP) of the NCBI contains extensive information on single nucleotide variants in every gene sequence. This database has been utilized to gather important BMP2 and BMP4 gene variations and their rs IDs. SNPs were extracted from Ensembl genome browser using the Chicken genome (GRCg6a; http://asia.ensembl.org/Gallus_gallus/) (BMP2-ENSGALG00000029301 and BMP4-ENSGALG00000012429). To find the most detrimental SNPs, in silico harmful SNP prediction algorithms were applied. Among these techniques were the sorting intolerant from tolerant (SIFT) [22], polymorphism phenotyping v2 (PolyPhen-2) [23], consensus deleteriousness score for missense mutations (Condel), M-CAP, MutPred, Mutation Assessor, and protein variation effect analyzer [24]. PolyPhen-2 uses the Nave Bayes approach to determine the functional significance of an allele change and its effect on the population [23]. PolyPhen-2 prediction is highly dependent on the number of sequences, their phylogeny, and the structural properties of the substitution [25]. The MutPred tool can classify an amino acid alteration as detrimental/disease-associated or neutral. This program examines three types of attributes: evolutionarily conserved amino acid sequences, protein structure and dynamics, and atomic and molecular alterations caused by amino acid substitutions [26]. PROVEAN is a sequence-based prediction tool that quantifies the effect of variation in protein sequences on function [27]. The effect of harmful nsSNPs in the protein sequence was quantified using delta alignment scores based on the variant version and reference protein sequence [28]. The PhD-SNP software was used to investigate how protein function is altered by mutations [29]. Evolutionary information distinguishes the neutral protein's SNPs associated with Mendelian and complex diseases [30]. The I-mutant3.0 predictor uses the support vector machine (SVM) approach to determine the change in stability induced by a single-site mutation based on the structure or sequence of a protein [31]. The mutant's DDG (kcal/mol) and RI are calculated using I-mutant3.0 (reliability index). SNAP2 predicts the effect of mutations on protein function through a neural network [32].

### 2.3. Conservation and Post-Translation Modification Sites Prediction

The ConSurf online tool was used to analyze the native BMP2 and BMP4 proteins [33, 34]. This online tool examines the evolutionary pattern of macromolecule amino acid or the nucleic acid (DNA/RNA) changes among homologous sequences to identify the areas crucial for the structure and function [35, 36]. The conservation scores from the protein sequence were calculated by utilizing the Bayesian computation technique. For further analysis, the nsSNP identified in the highly conserved area were also evaluated. A score of 1–4 was deemed changeable, whereas 5–6 and 7–9 were considered intermediate and conserved, respectively. The ModPred service (http://www.modpred.org/) was used to predict post-translational modification sites within the chicken BMP sequences. It is a sequence-based predictor of proteins' PTM (post-translational modification) sites. The server comprises 34 ensembles of logistic regression models; each was trained independently a cluster of 126,036 non-redundant experimentally confirmed sites for 23 different polymorphisms culled from Adhoc literature and public sources [37].

### 2.4. 3D Protein Modelling and Structural Analysis

The crystal structures of chicken BMP2 and BMP4 were generated with the web applications Phyre2 (http://www.sbg.bio.ic.ac.uk/phyre2/html) and the Swiss model (http://swissmodel.expasy.org) [38, 39]. Based on the phylogenetic connection between the sequences and utilizing the bioinformatics tool, ConSurf server (http://consurftest.tau.ac.il) [40, 41], the amount of evolutionary conservation of amino acid/nucleic acid locations in the protein was predicted. The homology modelling approach was used to estimate the structure of chicken BMP2 and BMP4. The I-TESSAR and Swiss modelling methods [36, 42] were used to predict the 3D structures of wild-type and mutant BMP2 and BMP4. The MolProbity server was employed to validate the structures of all the predicted models [43]. This server predicts protein structure using MODELLER v8.2 and use *Z*-score to categorize the protein sequence as excellent (*Z* − score > 7.5) or poor (*Z* − score < 7.5) [44]. The HOPE project, which uses UniProtKB and DAS servers to give 3D structural visualization to the mutant proteins, was extended further [45].

### 2.5. Prediction of the Protein Ligand-Binding Site in nsSNP

In this study, the FTSite server, an energy-based approach that correctly identifies the binding sites of around 94% of the apoproteins from two test sets, was used to find alternative binding site prediction methods [44, 46, 47]. Protein data bank (PDB) file of BMP2 and BMP4 protein structure was used to anticipate the binding locations. The COACH and I-Tasser Internet servers were utilized to identify the binding sites [34, 42]. The ligand-binding targets were predicted with the help of COACH server that uses two comparative methods, TM-SITE [46, 48] and S-SITE. The BioLiP protein function database is utilized in these methods to recognize ligand-binding sites [44, 49]. To predict the final ligand-binding site of the protein, PDB structures of the wild and mutant BMP proteins were submitted to the server for analysis.

## 3. Results

### 3.1. Retrieval and Distribution of SNPs

SNPs were extracted from the Ensembl genome browser using the Chicken genome (GRCg6a; http://asia.ensembl.org/Gallus_gallus/) (BMP2-ENSGALG00000029301 and BMP4-ENSGALG00000012429) and retrieved 5 SNPs in the 3′UTR area, 8 SNPs in the 5′UTR region, 57 SNPs in the noncoding region, and 11 missense variations in chicken BMP2 gene. The BMP4 gene contains 24 SNPs in the noncoding region and 18 missense variations. These 11 missense mutations of BMP2 and 18 missense mutations of BMP4, or nsSNP, were submitted to various SNP prediction tools to find out their effect. This resulted in a classification of nsSNP as either neutral or neutral detrimental to the structure and function of the BMPs (Table 1; Table 2). In the current study, only the nsSNP were further analyzed since their variations can encode a protein's function or structure. Each transcript (i.e., splice isoform) for the given gene is shown in the variation image and any related variation. The effects on the transcript (if any), position in genomic coordinates, alleles, encoded amino acids, and amino acid coordinates (if any) are all mentioned. The variant's source (or sources) and the validation status are also displayed. This information is graphically represented in the variation picture (Figure 1). With the inclusion of protein domains mapped to amino acid sequences, any protein structure and function changes may be estimated.

### 3.2. Evolutionary History of Genes

Using gene families, evolved from a common ancestor to demonstrate the evolutionary history of gene families, BMP2 and BMP4 gene trees were constructed. By reconciling the gene tree with the species tree, it is possible to infer orthologues and paralogues across the two gene trees. This allows us to distinguish between duplication and speciation processes. There is a clear agreement with reciprocal best methods in the basic instance of orthologous genes that are distinct. On the other hand, the gene tree pipeline can discover more complicated one-to-many and many-to-many relationships (Figure 2). The number of birds (chicken) to mammal orthologues increases considerably due to this, and the number of birds/mammal or fly/mammal orthologous gene predictions increases even more dramatically as a result. Using this technique, we may also predict “time” duplication occurrences that result in paralogues by determining the most recent common ancestor (i.e., taxonomy level) for a particular internal node of the tree. The consensus topology was made up of clades that have been identified in any of the input trees. Phyml with the HKY model was utilized to estimate the branch lengths based on the DNA alignment and then used to construct the final consensus tree (Figure 2). Multiple alignments of the peptides (green bars) were generated. Green bars represent areas of amino acid alignment, whereas white bars represent gaps in the alignment. Consensus alignments are indicated by dark green bars.

### 3.3. Functional Consequence of nsSNP

The single nucleotide variations of the BMP2 and BMP4 genes, obtained using dbSNP analysis, were submitted for the computational analysis utilizing several software tools. SIFT, PolyPhen-2, I-Mutant, PHD-SNP, and PROVEAN were among the methods employed to predict SNPs in silico (see Tables 1 and 2). Because of sequence homology, the SIFT method has been used to assess the influence of amino acid replacement on the protein function. Because these algorithms used different criteria to evaluate whether an nsSNP was detrimental or neutral, the percentages of harmful and neutral nsSNP in BMP2 and BMP4 have been summarized in Table 1. According to the SIFT results, 10 SNPs were deleterious, and only one was found to be tolerated in BMP2, while in BMP4, out of 18 SNPs, 12 were harmful and six were tolerated. To improve the accuracy of computational methods, the PolyPhen-2, I-Mutant, PHD-SNP, and PROVEAN tools were used to validate SNPs predicted in SIFT (Tables 1 and 1). Out of 11 SNPs submitted to PolyPhen-2 analysis, nine were projected to be probably harmful, and two were identified to be benign in BMP2. For BMP4, out of 18 SNPs, 14 were possibly harmful, and 4 were found to be benign (Tables 1 and 2). PolyPhen-2 calculates PSIC (position-specific independent score) for each input variable. PHD-SNP predicted all SNPs as diseased in BMP2, while seven were neutral in BMP4. The I-Mutant analysis demonstrates that all potential nsSNP, except one, decreased BMP2 and BMP4 activity by lowering its stability to DDG > 0.5 Kcal/mol. For further analysis, SNPs were submitted to PROVEAN analysis; eight were projected to be harmful, whereas three were predicted to be neutral. Predicted all SNPs as diseased in BMP4 and 12 SNPs as diseased, while six were neutral in BMP4 (Tables 1 and Table 2).

### 3.4. Structure Modelling and Domain Prediction

Interpro and the NCBI Conserved Domain Search program projected that BMP2 and BMP4 proteins include a large domain conserved across species. TGF-beta is the domain which contains amino acids 275–392 and was discovered in 1998. The capacity of proteins to execute various tasks or interact with other molecules depends on their tertiary structural composition [50]. RAMPAGE was used to evaluate the stability of BMP2 and BMP4 model protein structures that contained nsSNP (Figure 3 for the wild and mutated type BMP2 model protein structure and Figure 4 for the wild and mutated BMP4 model structure). To broaden the scope of these studies, we computed the root mean square deviation (RMSD) and the Tm-score for the high-risk nsSNP. The average distance between the alpha carbon backbones of wild type and mutant protein models is evaluated by the RMSD. In contrast, the topological similarity between wild type and mutant protein models is determined by the Tm-score. When the RMSD is large, the mutant structure differed from the wild-type structure. In addition, our finding suggests that the high-risk nonsynonymous SNPs have a substantial impact on the structural stability of the TGF-beta domain of these proteins.

### 3.5. Conservation and Post-Translational Modification Sites

In a biological system, proteins containing conserved amino acids are involved in various cellular processes, including genome stability [51]. Amino acids that occupy enzyme sites or required for protein-protein interaction are more conserved in proteins than other amino acids in the same molecule [52]. As a result, nsSNP located in conserved parts of the protein are more harmful than nsSNP located in variable sections of the protein. The evolutionary conservation profile of the BMP2 and BMP4 genes was predicted by using the ConSurf web browser. This browser uses Bayesian techniques to detect functional and structural residues and assess evolutionarily conserved amino acid residues in the proteins. This data was used to examine the possibility of high-risk nsSNP in the proteins BMP2 and BMP4 to cause damage. ConSurf analysis showed ten highly conserved amino acid residues in the TGF-beta-domain of the BMP2 and BMP4. The evolutionary information is used to detect if a change in an amino acid would affect the activity of the protein. The conservation score of amino acid residues in the BMP2 and BMP4 proteins was determined using the ConSurf web service, which was then used to investigate the potential effects of 11 and 18 nonsynonymous single nucleotide polymorphisms predicted by different computational tools in BMP2 and BMP4, respectively.

The anticipated function or structure of highly conserved residues is determined by the position of the residues on the protein surface vs within the protein's core. However, we only looked at residues whose locations corresponded to those of seven high-risk nsSNP that we had found. Considering this, nsSNP situated at these conserved areas are extremely detrimental to protein function compared to those at nonconserved locations. According to the results of ConSurf, the residues Y316S, V386G, E387G, C389G, and C391G nsSNP in the BMP2 and H344P, S347P, and V357A nsSNP in BMP4 are well conserved with a conservation score of nine. The mutant residue is smaller, which may result in interaction loss. At this location, the mutation introduces a more hydrophobic residue. This can result in the breakdown of hydrogen bonds and the disruption of proper folding. The average conservation of four amino acids was anticipated (Figures 5 and 6 and Tables 3 and 4).

### 3.6. Ligand-Binding Site Prediction

The FTSite server projected that the BMP2 and BMP4 contain three binding sites. The first binding site contained the residues L55, L58, T61, and G62, the second binding site at E145, V205, and T262, and the third binding site at positions E139 and L210 in BMP2 (Figure 7), while for BMP4, the first binding site contained the residues L53, G56, L63, and F66; the second binding site at A324, M379, Y381, D383, T262; and the third binding site at positions A49 and E52 (Figure 7). These binding sites were visualized by utilizing the PyMOL. Additionally, the COACH server predicted the ligand-binding sites (Table 5).

## 4. Discussion

BMPs are essential for the development of bone and cartilage, serving as the inspiration for the name of this protein family and the maintenance of normal bone function in adults. BMP signaling is required for various activities during early development, including cell proliferation, apoptosis, and differentiation [15]. BMPs also serve a critical role in maintaining adult tissue homeostasis, including preservation, vascular remodeling, and the fracture repair [53]. Any deficit in their production or function mostly results in a visible abnormalities or severe diseases in the tissues [54]. This study examined the functional implications with a functional assay that may be the most effective technique. Still, it is also the most expensive and time-intensive one available today. We have used a computational method to analyze SNPs in the BMP2 and BMP4 genes, employing various in silico techniques and diverse algorithms to understand the genes. The coding SNPs produce amino acid variation which affects the protein's function and increases the likelihood of developing an illness [55]. The nsSNP may not have a significant impact on protein function, and some may even have a neutral impact. As a result, to assess the susceptibility of particular SNPs to diseases, it is important to differentiate between harmful and neutral SNPs. Also essential is a concentrated effort to identify the SNPs responsible for the structural and functional implications of the BMP2 and BMP4 which are not yet been identified. However, employing a single bioinformatics tool to predict the pathogenic impact of an nsSNP may not be a valid method of prediction [56]. To predict BMP2 and BMP4 genetic variations, the following sequence and structure based tools were used: PolyPhen-2, SIFT, PROVEAN, MutPred, and PhD SNP. We subjected these 11 nsSNP mutations of BMP2 and 18 nsSNP mutations of BMP4, or nsSNP, to various SNP prediction methods, which resulted in a classification of nsSNP as either neutral or detrimental to the structure and function of the BMP proteins (Tables 1 and 2). We assessed the influence of the mutation on the following characteristics: the contacts formed by the mutated residue, the structural domains in which the residue is situated, changes to this residue, and known variations for this residue. Generally, mutation of a 100% conserved residue is detrimental to the protein [57]. However, the mutant residue has certain characteristics with the wild-type residue [58]. While this mutation may occur in very few instances, it is more likely detrimental to the protein. Numerous animal studies have established that the BMP superfamily is required for proper skeletal development and homeostasis [16, 59] and that BMP4 expression in bones is noticeable from the embryonic stage to the late adulthood in mice [60, 61]. Given the extensive phenotypic heterogeneity associated with BMP4 mutations [62], and the fact that BMP4 is expressed in bones [65], we sought to investigate the effects of BMP4 on the skeleton. The mutations in BMP2, that change a tyrosine to a serine at position 316, a valine to a glycine at position 386, a glutamic acid to a glycine at position 387, a cysteine to a glycine at position 389, and a cysteine to a glycine at position 391, all have distinct sizes, charges, and hydrophobicity values. These characteristics frequently change between the wild-type and the newly introduced mutant residues (Figure 3). Residues in the mutant are smaller than those in the wild type. The mutant and wild-type residues differ significantly. According to this conservation information, these mutations are almost certainly detrimental to the protein (Table 1). In case of BMP4, the change of a histidine into a proline at position 344, serine into a proline at position 347, and valine into alanine at position 357, the mutant residue is smaller than the wild-type residues (Figure 4). Also, the mutant residues are more hydrophobic than the wild-type residue (Table 2). The wild-type residues are annotated in UniProt as part of a cysteine bridge, which is critical for the protein's stability. Only cysteines can form these types of connections; the mutation abolishes this interaction, which has a detrimental effect on the 3D structure of the protein [63]. Along with the loss of the cysteine bond, the discrepancies between the old and new residues might result in structural instability [64].

A protein's tertiary structure determines how it interacts with the other biomolecules or performs distinct tasks. As a result, it is required to estimate the BMP2 and BMP4 gene's tertiary structure, as there is no crystal structure of chicken BMP2 and BMP4 proteins in the PDB. MUSTER was used to simulate the 3D structure. BMPs and mutant-type protein structures were subjected to energy reduction to determine their relative energies. The results revealed that the mutant type protein structure had lower total energy than the native type. There was a difference in total energy between the normal and mutant models following energy reduction of −10544.328 KJ/mol and −9734.687 KJ/mol. Mutation has a negative impact on protein stability, as evidenced by the mutant model having greater total energy. Project HOPE's 3D protein structure for BMP2 shows that the mutant residue is smaller than the wild-type residue, possibly indicating a reduction in the number of external contacts. There are also differences in the hydrophobicity between the wild-type and mutant proteins. The wild-type residue has a higher hydrophobicity than the mutant residue. With the FTSite technique, it is easy to pinpoint exactly where on the nsSNP binding took place. Understanding binding sites is essential since it is utilized in protein structure-based prediction, protein functional relationship determination, protein engineering, and medication development [65, 66]. The mutations are expected to be at a binding location and change the protein's ligand-binding affinity. Our findings imply that this illness-associated SNP should be regarded as a prominent reason behind BMP2 and BMP4 proteins malfunction, which may aid future research on the genetically inherited diseases. The 3D structure will serve as an excellent framework for the functional study of crystal structures obtained experimentally. As a result, SNPs in the protein may affect how it interacts with other molecules or parts of the protein. The in silico assay employed in this study enables critical, rapid, and low-cost evaluation of the biggest series of variations in BMPs that have been evaluated to date. This gives significant information that may be applied in a clinical practice. Thus, the current work demonstrates that a computational technique may be effectively used to identify the SNP targets by examining the effect of SNPs on the functional characteristics or molecular phenotype of a protein. These findings may contribute to a better understanding of the role of BMP SNPs in disease susceptibility.

## 5. Conclusions

Multidisciplinary study at several levels, including genomic and proteomic techniques and computational approaches, can help us comprehend the molecular pathways causing bone-related problems. The insight might contribute help develop sensible strategies for treating bone-related disorders. This study found that nsSNPs can affect BMP structure and function. It was predicted that five missense variations in the TGF-beta domain of chicken BMP2 and three in the TGF-beta domain of chicken BMP4 would be detrimental. There is a high risk of developing skeletal diseases such as ossification bones in chickens. Three of the most important SNPs were expected to be involved in post-translational variations out of the seven significant SNPs. As a result, these noncoding splice variants (nsSNPs) can be firmly regarded as significant candidates in the pathogenesis of skeletal disorders associated with BMP dysfunction. This will aid in discovering effective drugs and developing precision therapies. Wet lab experiments are necessary to determine the influence of these polymorphisms on the structure and function of the proteins. Also, understanding the pathogenesis of leg and skeletal abnormalities is important for better understanding the broiler leg illness. It is also important for reducing the economic loss caused by this disease, which is of considerable relevance and value.

## Figures and Tables

**Figure 1:** Graphical representation of the variations in BMP2 and BMP4 genes depicting all transcripts with variants mapping to each transcript shown by colored boxes.

**Figure 2:** The graph depicts the maximum likelihood phylogenetic tree that represents the evolutionary history of genes. These trees are compared with the species tree produced by TreeBeST. Internal nodes are marked for duplication (red boxes) or speciation (blue boxes). MUSCLE was used to do multiple alignments of the peptides (green bars). Green bars represent areas of amino acid alignment, whereas white bars represent gaps in the alignment. Consensus alignments are indicated by dark green bars.

**Figure 3:** The schematic representation of a wild type of chicken BMP2 including the TGF-beta domain and a mutant type produced using Phyre-2. Possible models were examined using Chimera and the PYMOL viewer. Each nsSNP in the TGF-Beta domain was assigned a potential 3D structure. Left side of each box represents the wild type's 3D structure, whereas the right side depicts the 3D structure of mutant type. Each mutant amino acid's location in mutated 3D structures and the wild type is marked in red, while the mutant amino acid's position is highlighted in blue.

**Figure 4:** The schematic representation of a wild type of chicken BMP4, including the TGF-beta domain and a mutant type, was produced using Phyre-2 version 2.0, which searches several sequence databases and constructs a 3D structure based on a homolog of a known structure. We examined possible models using Chimera and the PYMOL viewer. Each nsSNP in the TGF-beta domain was assigned a potential three-dimensional structure. Each box's left side represents the wild type's three-dimensional structure, whereas the right side depicts the mutant type's three-dimensional putative structure. Each mutant amino acid's location in mutated putative three-dimensional structures and the wild type is marked in red, while the mutant amino acid's position is highlighted in blue.

**Figure 5:** The color grade indicates the degree of the conservation status of amino acid residues. The grade (color) rises (1 is highly variable and 9 is a highly conserved site)—predictions of nsSNP in chicken-BMP2 show conservation profile by dotted rectangles.

**Figure 6:** The color grade indicates the degree of the conservation status of amino acid residues. The grade (color) rises (1 is highly variable and 9 is a highly conserved site)—predictions of nsSNP in chicken-BMP4 show conservation profile by dotted rectangles.

**Figure 7:** FTSite prediction, including ligand-binding sites. Zoom in on predicted ligand-binding sites using the FT site server; the pink, green, and blue colored meshes indicate the first, second, and third ligand-binding sites for BMP2 and BMP4 proteins, respectively.

**Table 1:** Prediction of functional outcomes of nsSNP in chicken BMP2.

					SIFT		Polyphen-2		I mutant			PHD-SNPs		PROVEAN	
Variant ID	Location	Alleles	Consequence	AA	Prediction	Score	Prediction	Score	SVM2 effect	DDG	RI	Effects	RI	Prediction	Score
rs737194602	3 : 15202267	A/C	Missense	C391G	Deleterious	0.00	Probably damaging	1.00	Decrease	-1.18	7	Disease	7	Deleterious	-9.47
rs732782874	3 : 15202273	A/C	Missense	C389G	Deleterious	0.00	Probably damaging	1.00	Decrease	-1.39	8	Disease	8	Deleterious	-9.521
rs740973105	3 : 15202278	T/C	Missense	E387G	Deleterious	0.01	Probably damaging	1.00	Decrease	-1.24	8	Disease	7	Deleterious	-4.975
rs734280202	3 : 15202281	A/C	Missense	V386G	Deleterious	0.00	Probably damaging	1.00	Decrease	-2.51	10	Disease	7	Deleterious	-5.58
rs734737781	3 : 15202491	T/G	Missense	Y316S	Deleterious	0.00	Probably damaging	1.00	Decrease	-1.31	7	Disease	7	Deleterious	-8.503
rs732058165	3 : 15202764	T/C	Missense	E225G	Deleterious	0.00	Probably damaging	1.00	Decrease	-1.36	7	Disease	4	Deleterious	-5.567
rs316999343	3 : 15202860	A/C	Missense	V193G	Deleterious	0.00	Probably damaging	1.00	Decrease	-2.57	9	Disease	8	Deleterious	-6.097
rs731854940	3 : 15202944	T/G	Missense	H165P	Deleterious	0.00	Probably damaging	1.00	Increase	0.07	5	Disease	8	Deleterious	-4.168
rs739775323	3 : 15202996	T/G	Missense	I148L	Tolerated	1.00	Benign	0.001	Decrease	-0.15	0	Disease	1	Neutral	0.369
rs737097326	3 : 15202998	T/G	Missense	Q147P	Deleterious	0.01	Benign	0.343	Decrease	-0.22	3	Disease	8	Neutral	-2.298
rs739140582	3 : 15203003	T/G	Missense	E145D	Deleterious	0.02	Probably damaging	0.62	Decrease	-0.52	6	Disease	3	Neutral	-2.165

**Table 2:** Prediction of functional outcomes of nsSNP in chicken BMP4.

					SIFT		PolyPhen-2		I-Mutant			PHD-SNPs		PROVEAN	
Variant ID	Location	Alleles	Consequence	AA	Prediction	Score	Prediction	Score	SVM2 effect	DDG	RI	Effects	RI	Prediction	Score
rs737608757	5 : 58714930	A/G	Missense	V357A	Deleterious	0.00	Probably damaging	0.997	Decrease	-1.77	9	Disease	9	Deleterious	-3.648
rs732839481	5 : 58714961	A/G	Missense	S347P	Deleterious	0.00	Probably damaging	0.988	Decrease	-0.15	3	Disease	7	Deleterious	-3.817
rs734844742	5 : 58714969	T/G	Missense	H344P	Deleterious	0.00	Probably damaging	1.00	Decrease	0.13	3	Disease	5	Deleterious	-9.096
rs741287624	5 : 58715180	T/G	Missense	T274P	Deleterious	0.00	Probably damaging	1.00	Decrease	-0.65	7	Disease	2	Deleterious	-5.855
rs730990074	5 : 58715182	A/G	Missense	V273A	Deleterious	0.00	Probably damaging	0.909	Decrease	-1.64	9	Disease	6	Deleterious	-3.59
rs313051524	5 : 58715219	A/G	Missense	Y261H	Tolerated	0.11	Benign	0.005	Decrease	-1.2	6	Disease	7	Neutral	1.491
rs317399411	5 : 58715229	T/G	Missense	L257F	Deleterious	0.00	Probably damaging	1.00	Decrease	-1.23	7	Neutral	6	Deleterious	-2.543
rs740468830	5 : 58715281	A/G	Missense	L240P	Tolerated	0.42	Probably damaging	0.998	Decrease	-0.97	4	Neutral	6	Neutral	-0.595
rs731863862	5 : 58715333	A/C	Missense	W223G	Deleterious	0.00	Probably damaging	1.00	Decrease	-2.36	9	Disease	7	Deleterious	-11.743
rs738054003	5 : 58715355	A/C	Missense	D215E	Deleterious	0.00	Probably damaging	0.985	Decrease	-0.15	5	Neutral	2	Deleterious	-3.895
rs739999946	5 : 58715369	A/C	Missense	W211G	Deleterious	0.00	Probably damaging	1.00	Decrease	-2.16	9	Disease	8	Deleterious	-11.404
rs731128170	5 : 58715486	A/C	Missense	W172G	Tolerated	0.36	Probably damaging	0.865	Decrease	-1.92	9	Neutral	7	Neutral	0.94
rs738537703	5 : 58715503	T/C	Missense	E166G	Tolerated	0.19	Benign	0.001	Decrease	-1.09	7	Neutral	7	Neutral	-1.046
rs739516377	5 : 58715506	A/C	Missense	V165G	Deleterious	0.04	Probably damaging	0.99	Decrease	-1.63	7	Neutral	1	Deleterious	-3.592
rs313359121	5 : 58715596	A/G	Missense	V135A	Tolerated	0.45	Benign	0.001	Decrease	-1.95	9	Neutral	7	Neutral	0.55
rs733650353	5 : 58716514	A/G	Missense	F120S	Deleterious	0.00	Probably damaging	0.999	Decrease	-1.68	8	Disease	6	Deleterious	-5.932
rs741393694	5 : 58716530	T/G	Missense	N115H	Deleterious	0.00	Probably damaging	1.00	Decrease	-0.67	8	Disease	0	Deleterious	-3.673
rs317497962	5 : 58716842	T/G	Missense	I11L	Tolerated	1.00	Benign	0.001	Decrease	-0.71		Neutral	7	Neutral	0.442

**Table 3:** Predictions of nsSNP in chicken-BMP2 presenting conservation pattern and their post-translational sites.

SNP ID	Variants	Conservation score	B/E	F/S	PTM
rs737194602	C391G	9	E	F	Proteolytic cleavage
rs732782874	C389G	9	B	S	—
rs740973105	E387G	9	E	F	Proteolytic cleavage
rs734280202	V386G	9	B	S	—
rs734737781	Y316S	9	B	S	Proteolytic cleavage
rs732058165	E225G	9	B	—	Amidation
rs316999343	V193G	9	B	—	—
rs731854940	H165P	7	B	—	Proteolytic cleavage
rs739775323	I148L	6	B	—	—
rs737097326	Q147P	8	E	F	—
rs739140582	E145D	9	E	F	Amidation, sulfation

B: buried; E: exposed; F: functional; S: structural; PTM: post-translation modification sites.

**Table 4:** Predictions of nsSNP in chicken-BMP4 presenting conservation pattern and their post-translational sites.

SNP ID	Variants	Conservation score	B/E	F/S	PTM
rs737608757	V357A	9	B	S	Proteolytic cleavage
rs732839481	S347P	9	E	F	Proteolytic cleavage
rs734844742	H344P	9	E	F	Proteolytic cleavage
rs741287624	T274P	9	B	S	—
rs730990074	V273A	8	B	S	Proteolytic cleavage
rs313051524	Y261H	1	E	—	—
rs317399411	L257F	6	B	—	Proteolytic cleavage
rs740468830	L240P	2	E	—	—
rs731863862	W223G	9	B	S	—
rs738054003	D215E	1	E	—	Proteolytic cleavage
rs739999946	W211G	7	B	—	—
rs731128170	W172G	1	E	—	—
rs738537703	E166G	2	E	—	—
rs739516377	V165G	4	B	—	Proteolytic cleavage
rs313359121	V135A	1	E	—	—
rs733650353	F120S	9	B	—	—
rs741393694	N115H	9	E	F	Proteolytic cleavage
rs317497962	I11L	6	B	—	Proteolytic cleavage

B: buried; E: exposed; F: functional; S: structural; PTM: post-translation modification sites.

**Table 5:** Prediction of ligand-binding sites within BMP2 and BMP4 proteins using COACH.

BMP2	COACH results			
	C-score	Cluster size	Ligands name	Predicted binding residue
	0.16	10	ZN	321, 325, 389, 391
	0.03	2	MG	145, 205, 262
	0.03	2	NAG	205, 207, 208, 211
	0.03	2	NI	58, 60, 348
	0.03	2	EDO	3, 6
	0.02	1	ZN	152, 232
	0.02	1	MG	300, 301
	0.02	1	PEPTIDE	354, 355, 356, 382, 392
	0.02	1	PEPTIDE	79, 82
	0.02	1	MG	56, 390
	TM-site			
	C-score	Cluster size	Ligands name	Predicted binding residues
	0.18	2	Mg(1), ZN(1)	321, 325, 389, 391
	0.15	1	Mg(1)	300, 301
	0.13	1	C8E(1)	369, 377
	0.12	2	T55(1), EDO(1)	3, 6
	0.12	1	Mg(1)	145, 205, 262
	S-site			
	C-score	Cluster size	Ligands name	Predicted binding residues
	0.32	9	Zn, FE, UUU	292, 294, 321, 325, 354, 355, 356, 357, 389, 391
	0.11	1	DIO	7, 309, 369
BMP4	COACH results			
	C-score	Cluster size	Ligands name	Predicted binding residues
	0.1	6	ZN	333, 337, 368, 369
	0.05	3	Nuc.Acid	53, 56
	0.05	3	SIA	320, 322, 324, 325, 326
	0.03	2	k-mer	304, 306, 344, 346, 401
	0.03	2	CA	312, 313
	0.03	2	UNK	380, 382
	0.02	1	PEPTIDE	366, 367, 368, 394, 404
	0.02	1	N/A	113, 303, 304, 337, 340, 344, 346, 347, 356, 357
	0.02	1	BU2	116, 159, 269
	0.02	1	MAL	325, 378, 380, 392
	TM-site			
	C-score	Cluster size	Ligands name	Predicted binding residues
	0.17	2	CA	312, 315
	0.15	3	NUC, MPG	53, 56
	0.13	1	UNK	380, 382
	0.13	1	EQU	393, 394
	0.12	1	CLA	62, 66
	S-site			
	C-score	Cluster size	Ligands name	Predicted binding residues
	0.32	9	ZN, III, FE	304, 333, 344, 346, 366, 367, 368, 369, 394, 401
	0.11	1	DIO	319, 321, 381

## Data Availability

The data relating to this article will be available openly to the readers.

## Abbreviations

BMPs: Bone morphogenetic proteins
TGF: Transforming growth factor
nsSNP: Single-nucleotide polymorphisms
MSCs: Mesenchymal stem cells
GDF: Growth differentiation factor
TD: Tibial dyschondroplasia
NCBI: National Center for Biotechnology Information
SIFT: Sorting intolerant from tolerant
SVM: Support vector machine
RMSD: Root mean square deviation.
